The article "Protective Effect of Rifampicin Loaded by HPMA-PLA Nanopolymer on Macrophages Infected with Mycobacterium Tuberculosis" was retracted in 2023. Reasons: unreliable results or conclusions; concerns about the data; concerns about the peer review; concerns about the citations.

# Protective Effect of Rifampicin Loaded by HPMA-PLA Nanopolymer on Macrophages Infected with Mycobacterium Tuberculosis

**DOI:** 10.1155/2022/5784283

**Published:** 2022-01-04

**Authors:** Guoping Yang, Guofu Wang, Liting Liu, Kaixin Zhai, Xiaowen Chen, Yue Chen, Lixian Wu

**Affiliations:** Department of Medical Microbiology and Immunology, Clinical Molecular Immunology Innovation Team, Dali University, Dali, 671000 Yunnan, China

## Abstract

**Purpose:**

This research was designed to investigate the protective effect of rifampicin (RIF) loaded by N-(2-hydroxypropyl) methylacrylamide- (HPMA-) polylactic acid (PLA) nanopolymer on macrophages infected with Mycobacterium tuberculosis (MTB).

**Methods:**

We first induced H37Rv to infect macrophages to build a cell model. Then, the HPMA-PLA nanopolymer loaded with RIF was prepared to treat MTB-infected macrophages. The macrophage activity was tested by the 3-(4,5-dimethylthiazol-2-yl)-2,5-diphenyltetrazolium bromide (MTT) assay, the nitric oxide (NO) in cells was measured through Griess reagent, and the bacterial activity of MTB was observed via the colony-forming unit (CFU) assay. The inflammation-related factors in cells were detected via the enzyme-linked immunosorbent assay (ELISA), the apoptosis of macrophages was examined via flow cytometry, and the expression of apoptosis-related proteins was determined by western blot (WB).

**Results:**

HPMA-PLA had no obvious toxicity to macrophages. The expression of NO and inflammatory factors in macrophages infected with MTB increased significantly, but the apoptosis rate was not significantly different from that of uninfected cells. However, after treatment with HPMA-PLA-RIF or free RIF, the inflammatory reaction of infected cells was inhibited, the expression of NO was decreased, the apoptosis rate was increased, and the bacterial activity in cells was decreased, with statistically significant differences; moreover, HPMA-PLA-RIF was more effective than free RIF.

**Conclusions:**

HPMA-PLA-RIF has a high protective effect on macrophages infected with MTB, with high safety. Its protective mechanism is at least partly through inhibiting the production of NO and inflammatory response, which can inhibit bacterial activity and induce cell apoptosis.

## 1. Introduction

Tuberculosis (TB) is a global infectious disease caused by a latent infection of the Mycobacterium tuberculosis (MTB) that attacks the host's immune system in an attempt to activate the infection, a disease caused by the bacterium. According to the World Health Organization (WHO), approximately 1.5 million people died from TB in 2018 [1]. Despite the continuous advances in medical technology and the development of vaccines, the morbidity of TB has not been significantly improved, posing a serious threat to human life and health [2, 3]. Rifampicin (RIF) is one of the drugs approved for the treatment of TB at present. Although it plays a certain role in reducing the mortality of TB, its low targeting of macrophages leads to a low killing rate, resulting in a longer treatment cycle for patients as well as some inevitable toxic and side effects [4, 5]. Therefore, more efficient and active killing of MTB in macrophages and reducing the emergence of drug-resistant MTB are the most pressing challenges facing TB treatment [6]. This study will also contribute to the treatment of TB, hoping to provide some reference for the effective treatment of TB patients from the breakthrough point of the nanotargeted drug delivery system.

The article "Protective Effect of Rifampicin Loaded by HPMA-PLA Nanopolymer on Macrophages Infected with Mycobacterium Tuberculosis" was retracted in 2023. Reasons: unreliable results or conclusions; concerns about the data; concerns about the peer review; concerns about the citations.

With the development of nanotechnology in recent years, its application in the medical field is becoming more and more extensive, among which the nanodrug delivery system is one of the more representative applications [7]. But for TB, how to develop a nanotargeted drug delivery system to effectively target MTB in macrophages is still a huge challenge [8]. N-(2-Hydroxypropyl) methacrylamide (HPMA) is a hydrophilic copolymer, which can improve the solubility of hydrophobic drugs in water. In view of its ability to prepare nanopolymer micelles, we also choose it as a hydrophilic carrier [9]. The main advantages of copolymer micelles are that they are readily bound by a variety of chemical species and are an important and attractive class of drug carriers for intravenous administration of hydrophobic drugs [10]. Polylactic acid (PLA) has good biocompatibility and biodegradability and can effectively encapsulate hydrophobic drugs [11], so we chose it to combine with HPMA to load RIF.

In this study, the HPMA-PLA nanopolymer loaded with RIF was prepared and applied to macrophages infected with MTB, to observe its effects on cells.

## 2. Materials and Methods

### 2.1. Synthesis and Characterization of RIF-Loaded HPMA-PLA Nanopolymer

First, HPMA was synthesized referring to the method in the previous literature [12]. Totally, 1 g anhydrous sodium sulfate (11.9 mmol/g) and 0.85 g 1-aminopropane-2-alcohol were dissolved in dichloromethane (DCM) and cooled at 0°C. Methacryloyl chloride was added drop by drop into DCM under cooling and intense agitation for 1 h. The mixture was then stirred again for 30 min. Then, at 15°C, anhydrous sodium sulfate was added, and the mixture was filtrated and dried. HPMA was obtained from DCM by crystallization at -20°C, and pure HPMA was gained by recrystallization. Totally, 500 mg PLA (0.05 mmol/mg) and 7 mg HPMA (0.05 mmol/mg) were dissolved in 5 mL DCM and stirred mixed for 24 h to obtain the HPMA-PLA copolymer. The RIF-loaded HPMA-PLA nanocopolymer was prepared by the direct dissolution method, in short, by adding two solutions to suitable drug polymers. Besides, 10 mg RIF was dissolved in ethanol and dropped into the distilled water solution dissolved with HPMA-PLA. The solution mixture was thoroughly stirred and fused at room temperature for 24 h to synthesize HPMA-PLA-RIF. The characterization of HPMA-PLA-RIF, including size analysis, dispersion index, and surface morphology, was detected by using a scanning electron microscope (SEM).

The article "Protective Effect of Rifampicin Loaded by HPMA-PLA Nanopolymer on Macrophages Infected with Mycobacterium Tuberculosis" was retracted in 2023. Reasons: unreliable results or conclusions; concerns about the data; concerns about the peer review; concerns about the citations.

### 2.2. Cell Culture and Infection

The mouse macrophage cell line J774A.1, purchased from the National Center for Cell Science Center (NCCS, Pune), was stored in Dulbecco's modified Eagle medium (DMEM) containing 10% fetal calf serum (FCS; complete medium). Before infection, the culture was suspended in antibiotic-free DMEM, and a Probe Sonicator was used to conduct ultrasonic treatment (amplitude: 10%) with a Probe Sonicator with three pulses of 10 s each, to destroy bacterial aggregation and obtain a uniform suspension. The bacterial suspension was then centrifuged at 400 × *g* for 5 min. After centrifugation, 1.5 mL of the suspension was collected to determine the optical density (OD) by spectrophotometry at 600 nm. In a humid CO_2_ incubator at 37°C and 5% CO_2_, the cells were inoculated on a 96-well plate at 0.1 × 10^6^ cells/well. Those exposed to H37Rv with a multiplicity of infection (MOI) of 10 for 3 h were included in the H37Rv group. A control group without infection was set up. Extracellular bacteria were eliminated by removing the supernatant and washing adhered cells with Hanks' balanced salt solution (HBSS). Adhered J774 cells (1 × 10^5^ per well) infected with MTB H37Rv were then exposed to 10 g/mL HPMA-PLA-RIF or 10 g/mL RIF for 24 h, respectively, as the H37Rv+HPMA-PLA-RIF group and H37Rv+RIF group.

### 2.3. Assay of Nitric Oxide (NO) and Inflammatory Factors

The concentration of NO was measured using the Griess reagent (Promega, USA). J774 cells infected with MTB were exposed to 10 *μ*g/mL HPMA-PLA-RIF for 24 h and centrifuged at 400 × *g* for 8 min to remove the cells and collect the supernatant. Meanwhile, the nitrite standard was prepared by diluting 100 *μ*M nitrite solution to 0.39 *μ*M through double dilution. Totally, 50 *μ*L cell-free supernatant and nitrite standard solution were added to the 96-well tissue culture plate. Then, 50 *μ*M sulfanilamide solution was added to each well and incubated at room temperature for 20 min, followed by the addition of 50 *μ*M N-1-naphthylethylenediamine hydrochloride for 10 min of incubation. The absorbance was measured at 540 nm using a Victor™×3 Multilabel reader (PerkinElmer 2030). The tumor necrosis factor-*α* (TNF-*α*) and interleukin-6 (IL-6) levels were detected by ELISA.

The article "Protective Effect of Rifampicin Loaded by HPMA-PLA Nanopolymer on Macrophages Infected with Mycobacterium Tuberculosis" was retracted in 2023. Reasons: unreliable results or conclusions; concerns about the data; concerns about the peer review; concerns about the citations.

### 2.4. 3-(4,5-Dimethylthiazol-2-yl)-2,5-diphenyltetrazolium Bromide (MTT) Assay

The MTT assay was used to determine the toxicity of HPMA-PLA to macrophages and the effect of HPMA-PLA-RIF on the proliferation of J774 cells infected with H37Rv. J774 cells were inoculated into the Roswell Park Memorial Institute- (RPMI-) 1640 (Thermo Fisher Scientific) medium on the 96-well plate at a density of 1 × 10^4^ cells/well and incubated at 37°C with 5% CO_2_ in air for 24 h. Next, the cells were treated with 100 *μ*L freshly prepared HPMA-PLA-RIF and further cultured at 37°C with 5% CO_2_ for 48 h. For the MTT assay, 20 *μ*L MTT solution was supplemented and cultivated for 5 h; then, 100 *μ*L DMSO (dimethyl sulfoxide) was added and the plate was placed on an oscillator for 5 min. Then, the maximum absorbance was measured at 590 nm and the cell viability was calculated.

### 2.5. Apoptosis Assay

Cell death was quantified via flow cytometry and fluorescence microscopy with propidium iodide (PI). J774 cells were inoculated into a 6-well plate at a density of 1.6 × 10^6^ cells/well. The cells were then washed with phosphate buffer solution (PBS) and then immobilized in cold methanol at -20°C for 2 h. The fixed cells were treated with RNase (20 *μ*g/mL) and dyed with PI at room temperature in the dark for 30 min. Thereafter, PI fluorescence of mononuclear cells was measured using flow cytometry (BD FACSCalibur, Becton Dickinson, USA). The data were analyzed by using CellQuest Pro V 3.2.1.

### 2.6. Apoptosis-Related Proteins Are Tested by WB

Proteins in cells were extracted with Radioimmunoprecipitation Assay (RIPA) lysis buffer, centrifuged (16,000 × *g*, 4°C) for 10 min, and stored at -80°C. The protein concentration was determined by the bicinchoninic acid (BCA) assay. Then, 30 *μ*g proteins in each group was analyzed using 10% sodium dodecyl sulfate-polyacrylamide gel electrophoresis (SDS-PAGE). Subsequently, the protein was transferred to the polyvinylidene fluoride (PVDF) membrane in a 100 V Bio-Rad TransBlot instrument (Bio-Rad Laboratories, Inc.). The membrane was then sealed with 5% nonfat milk powder for 2 h and incubated with the following primary antibodies at 4°C overnight: BCL2-associated X (Bax; 1 : 500; Sino Biological, Inc., Beijing, China, cat. no. 100787-T02), B-cell lymphoma-2 (Bcl-2; 1 : 500; Sino Biological, Inc., Beijing, China, cat. no. 10195-MM04T), and *β*-actin (1 : 1,000; Sino Biological, Inc., Beijing, China, cat. no. 100166-MM10). The next day, the membrane was washed with Tris-buffered saline and Tween (TBST) at room temperature three times for 5 min each and then incubated with the second antibody (goat anti-rabbit HRP; Taize Jiaye Technology Development Co., Ltd., Beijing, China, cat. no. 656120) for 2 h. After rinsing with PBS for 3 times (5 min each time) and absorbing the excess liquid, it was developed by electrochemiluminescence (ECL). ImageJ v1.4.9 software was used to quantify the relative protein expression of Bax, Bcl-2, and *β*-actin in the WB bands on each sample membrane, with *β*-actin as the internal reference.

The article "Protective Effect of Rifampicin Loaded by HPMA-PLA Nanopolymer on Macrophages Infected with Mycobacterium Tuberculosis" was retracted in 2023. Reasons: unreliable results or conclusions; concerns about the data; concerns about the peer review; concerns about the citations.

### 2.7. Intracellular Antinuclear Mycobacterium

J774 cells were inoculated into a 12-well tissue culture plate at 1 × 10^6^ cells/well and infected with MTB H37Ra with a MOI of 10 : 1 in the environment of 5% CO_2_ and 37°C. Four hours after infection, the cells were exposed to blank GP, soluble (pure) RB, or (RB-NP)-GP at equal concentration (10 *μ*g/mL). After that, macrophages were ablated in sterile water containing 0.025% (*w*/*v*) Triton X-100 at 0, 48, and 72 h after exposure. The lysate was continuously diluted (10× and 100×), in which 10 *μ*L was spread on a Middlebrooks 7H10 agar plate containing oleic acid-albumin-dextrose-catalase (OADC) supplement and cycloheximide. The plate was then incubated at 37°C under controlled humidity for 3 weeks. Finally, colony-forming units (CFU) were counted to determine the intracellular survival of MTB.

### 2.8. Statistical Methods

SPSS20.0 (EasyBio Technology Co., Ltd., Beijing, China) was used for statistical analysis, and Graphpad Prism 7.0 (Univ Biotechnology Co., Ltd., Shanghai, China) was used for image rendering and image export. The data in figures and tables were expressed as mean ± standard error of the mean (SEM). All data were analyzed using the *t*-test, and the comparisons among multiple groups were performed by one-way Analysis of Variance (ANOVA) and Bonferroni post hoc test, with the significance level set as *P* < 0.05.

## 3. Results and Discussions

### 3.1. Effect of HPMA-PLA-RIF on NO Production in Macrophages Infected with H37Rv

First, the characterization of HPMA-PLA-RIF was observed by SEM. The diameter of HPMA-PLA-RIF was 92.57 ± 1.33 nm, and the dispersion index was 0.483 ± 0.09 (Figure 1(a)). Subsequently, we observed the effect of HPMA-PLA-RIF on NO production in macrophages infected with H37Rv. It was found that compared with uninfected J774 cells, the NO production of J774 cells infected with H37Rv increased, with statistical significance (*P* < 0.05). After treatment with RIF or HPMA-PLA-RIF, the NO production of H37Rv-J774 cells decreased significantly, especially in the HPMA-PLA-RIF group, with statistical significance (*P* < 0.05) (Figure 1(b)).

The article "Protective Effect of Rifampicin Loaded by HPMA-PLA Nanopolymer on Macrophages Infected with Mycobacterium Tuberculosis" was retracted in 2023. Reasons: unreliable results or conclusions; concerns about the data; concerns about the peer review; concerns about the citations.

### 3.2. Effect of HPMA-PLA-RIF on Inflammatory Factors in Macrophages Infected with H37Rv

Compared with uninfected J774 cells, the levels of TNF-*α* (Figure 2(a)) and IL-6 (Figure 2(b)) were increased in J774 cells infected with H37Rv, with statistical significance (*P* < 0.05). After treatment with RIF or HPMA-PLA-RIF, the expression of TNF-*α* and IL-6 in H37Rv-J774 cells decreased, especially in the HPMA-PLA-RIF group, and the differences were statistically significant (*P* < 0.05).

### 3.3. Effect of HPMA-PLA-RIF on Proliferation of Macrophages Infected with H37Rv

First, HPMA-PLA was observed to have no obvious toxicity to infected or uninfected macrophages; that is, it had no significant effect on cell viability (*P* > 0.05, Figure 3(a)). Then, we treated H37Rv-J774 cells with RIF or HPMA-PLA-RIF and found that the macrophage viability infected with H37Rv was significantly inhibited, especially in those treated with HPMA-PLA-RIF, with statistical significance (*P* < 0.05, Figure 3(b)).

### 3.4. CFU Determination of Bacterial Activity of MTB

The bacterial activity of H37Rv-J774 cells was tested by the CFU assay. The results showed that H37Rv-J774 cells had obvious progressive growth of MTB compared with uninfected macrophages. After treatment with RIF or HPMA-PLA-RIF, the CFU count in H37Rv-J774 cells decreased significantly, and the decrease was more significant in the HPMA-PLA-RIF group, with statistical significance (*P* < 0.05) (Figure 4).

### 3.5. Effect of HPMA-PLA-RIF on Apoptosis of Macrophages Infected with H37Rv

The apoptosis of H37Rv-J774 cells was determined by flow cytometry (Figure 5(a)). The apoptosis rates of the control group, H37Rv group, H37Rv+RIF group, and H37Rv+HPMA-PLA-RIF group were 3.15 ± 0.68%, 31.47 ± 3.96%, 11.85 ± 1.63%, and 18.76 ± 1.99%, respectively. The results revealed no significant difference in the apoptosis rate between the H37Rv group and control group (*P* > 0.05). After intervention, it was found that compared with the H37Rv group, the apoptosis rate of H37Rv+RIF and H37Rv+HPMA-PLA-RIF groups increased significantly, with the highest found in the H37Rv+HPMA-PLA-RIF group, with statistical significance (Figure 5(b)) (*P* < 0.05).

### 3.6. Effect of HPMA-PLA-RIF on Apoptosis-Related Protein Expression in Macrophages Infected with H37Rv

Bax and Bcl-2 are key regulators of cell survival; the former can inhibit cell apoptosis, while the latter has the opposite effect, both of which play a crucial role in the apoptosis process of macrophages infected with H37Rv [13]. Therefore, in this study, we explored the effect of HPMA-PLA-RIF on the protein expression levels of Bax and Bcl-2 in macrophages infected with H37Rv by WB. It was found that there was no significant difference in the protein expression of Bax (Figure 6(a)) and Bcl-2 (Figure 6(b)) between the control group and the H37Rv group (*P* > 0.05). After treatment, the Bcl-2 expression in cells in H37Rv+RIF and H37Rv+HPMA-PLA-RIF groups was significantly lower than that in the H37Rv group, while the Bax expression was significantly higher than that in the H37Rv group, and the changes of cells in the H37Rv+HPMA-PLA-RIF group were more obvious than those in the H37Rv+RIF group, with statistical significance (*P* < 0.05).

The article "Protective Effect of Rifampicin Loaded by HPMA-PLA Nanopolymer on Macrophages Infected with Mycobacterium Tuberculosis" was retracted in 2023. Reasons: unreliable results or conclusions; concerns about the data; concerns about the peer review; concerns about the citations.

## 4. Discussion

Previously, RIF has been used as the first-line drug for TB and has shown certain efficacy against TB infection. However, with the emergence of extensive drug resistance involving a combination of multidrug resistance, the resistance of MTB to anti-TB drugs is getting stronger and stronger [14, 15]. Therefore, it is a major trend to develop better anti-TB treatment. In recent years, the continuous development of nanomedicine has opened up new ideas for the treatment of TB, in combination with nanotechnology that is widely used clinically. For instance, a study [16] has employed high-concentration (concentration ≥ 0.30 g/m) nanosilver combined with first-line anti-TB drugs as nanodrugs against the phagocytosis of MTB, and the results show that this treatment has a strong killing effect on drug-resistant strains of MTB.

In addition, more and more scholars have carried out *in vivo* and *in vitro* experiments on HPMA nanodelivery devices. Cheah et al. [17] found in their study that the application of HPMA nanodelivery devices loaded with doxorubicin in rats resulted in not only lower cardiovascular variability but also higher survival rate. Xiang et al. [18] reported that HPMA copolymer combined with cisplatin and digoxin can effectively promote immunogenic cell death and restore the immunogenicity of nonimmunogenic drugs. In this study, we successfully synthesized HPMA-PLA copolymer loaded with RIF, with the goal of improving the inhibitory effect of RIF on MTB by using nanopolymer as a carrier. As a new drug carrier, nanopolymer has been extensively used in recent years. For example, the HPMA-PLA copolymer loaded with bortezomib has been shown to be effective in the treatment of multiple myeloma [19]. HPMA as a hydrophilic shell layer and PLA as a hydrophobic core layer can form the HPMA-PLA polymer, while RIF is a hydrophobic drug. Because of the high content of polylactic acid in copolymer, RIF is encapsulated in micelles. And due to hydrophobic interaction, it is easily loaded into the hydrophobic core, with high drug solubility [20, 21]. Previous research [22] has shown that the formation of HPMA-PLA-RIF copolymer micelles enhanced the efficacy of drugs, improved the solubility of drugs, and combated the resistance of tuberculostatics. To observe whether HPMA-PLA has toxicity to macrophages, we intervened with infected or uninfected macrophages with HPMA-PLA without drug loading. The results showed that the activity of all macrophages did not change significantly, indicating that HPMA-PLA had no obvious toxicity to macrophages. Subsequently, the effect of HPMA-PLA copolymer micelles loaded with RIF on MTB was further investigated. HPMA-PLA-RIF was observed to significantly inhibit the bacterial activity of MTB, with higher efficacy than free RIF. This suggested that HPMA-PLA-RIF plays a good antibacterial role in macrophages infected with MTB.

The article "Protective Effect of Rifampicin Loaded by HPMA-PLA Nanopolymer on Macrophages Infected with Mycobacterium Tuberculosis" was retracted in 2023. Reasons: unreliable results or conclusions; concerns about the data; concerns about the peer review; concerns about the citations.

Some studies [23, 24] have reported that MTB infection can induce the release of IL-6 and TNF-*α*, as well as the production of NO by inducing nitric oxide synthase. The increased expression of inflammatory factors will further aggravate tissue damage, accompanied by drug resistance due to NO or other proinflammatory cytokines caused by emergency factors of the host [25, 26]. In our study, it was observed that the production of NO and the expression of IL-6 and TNF-*α* in macrophages infected with H37Rv increased significantly; however, their levels in cells decreased significantly after the intervention of RIF or HPMA-PLA-RIF, and the alleviation of inflammation was more significant in cells treated with HPMA-PLA-RIF. It indicates that HPMA-PLA-RIF can alleviate the inflammatory state of cells by inhibiting the production of NO and the expression of IL-6 and TNF-*α*, thereby exerting a protective effect against TB. Currently, it is known that MTB can be stored and replicated in macrophages, so apoptosis induction of macrophages infected with MTB is also a protective effect against MTB [27]. We further found that HPMA-PLA-RIF intervention could induce the apoptosis of macrophages infected with MTB, and its effect was stronger than that of free RIF. Consistent results were also obtained when detecting the expression of apoptosis-related proteins.

The novelty of this study is that the HPMA-PLA nanopolymer loaded with RIF has a protective effect superior to free RIF on H37Rv-infected macrophages by analyzing macrophage activity, NO release amount, inflammation-related factors, apoptosis, and apoptosis-related proteins, which provided a new theoretical basis for the treatment strategy of anti-TB drugs. However, there is still room for improvement in our research. First, animal experiments can be supplemented to verify the protective effect of HPMA-PLA-RIF in vivo. In addition, we can increase the research on HPMA-PLA-RIF-related molecular channels to further explore its potential mechanism of anti-infection. We will conduct supplementary studies from these two directions in the future.

The article "Protective Effect of Rifampicin Loaded by HPMA-PLA Nanopolymer on Macrophages Infected with Mycobacterium Tuberculosis" was retracted in 2023. Reasons: unreliable results or conclusions; concerns about the data; concerns about the peer review; concerns about the citations.

## 5. Conclusion

For TB patients, the existing treatments are not popular and are not good for patients because of their insignificant efficacy and long-term treatment process. On the contrary, the key advantages of nanocarriers such as nanopolymers can be utilized to address the shortcomings of existing chemotherapy approaches to treat MTB. This research is a preliminary attempt. Although it only reports *in vitro* experiments, the observational results clearly indicate its potential in anti-MTB drug delivery, which is worthy of further exploration.

## Figures and Tables

**Figure 1:** Effect of HPMA-PLA-RIF on NO production in macrophages infected with H37Rv. (a) Characterization of HPMA-PLA-RIF by SEM. (b) Effect of HPMA-PLA-RIF on NO production in macrophages infected with H37Rv. Note: ^∗^*P* < 0.05 and ^∗∗^*P* < 0.01*vs.* the control group; ^a^*P* < 0.05*vs.* the H37Rv group; ^b^*P* < 0.05*vs.* the H37Rv+HPMA-PLA-RIF group.

**Figure 2:** Effect of HPMA-PLA-RIF on inflammatory factors in macrophages infected with H37Rv. (a) The TNF-*α* expression. (b) The IL-6 expression. Note: ^∗^*P* < 0.05 and ^∗∗^*P* < 0.01*vs*. the control group; ^a^*P* < 0.05*vs*. the H37Rv group; ^b^*P* < 0.05*vs*. the H37Rv+HPMA-PLA-RIF group.

**Figure 3:** Effect of HPMA-PLA-RIF on proliferation of macrophages infected with H37Rv. (a) The toxicity of HPMA-PLA to macrophages. (b) Effect of HPMA-PLA-RIF on activity of macrophages infected with H37Rv. ^∗^*P* < 0.05.

**Figure 4:** CRU determination of bacterial activity of MTB. Note: ^∗^*P* < 0.05.

**Figure 5:** Effect of HPMA-PLA-RIF on apoptosis of macrophages infected with H37Rv. (a) Macrophage apoptosis detected by flow cytometry. (b) Comparison of the apoptosis rate. Note: ^∗^*P* < 0.05.

**Figure 6:** Effect of HPMA-PLA-RIF on apoptosis-related proteins in macrophages infected with H37Rv. (a) Western blot. (b) Bax protein expression. (c) Bcl-2 protein expression. Note: ^∗^*P* < 0.05.

## Data Availability

The labeled dataset used to support the findings of this study is available from the corresponding author upon request.
